# Multimodal Imaging under Artificial Intelligence Algorithm for the Diagnosis of Liver Cancer and Its Relationship with Expressions of EZH2 and p57

**DOI:** 10.1155/2022/4081654

**Published:** 2022-03-14

**Authors:** Yamin Zhang, Jie Cui, Wei Wan, Jinpeng Liu

**Affiliations:** ^1^Department of Oncology, Xi'an International Medical Center Hospital, Xi'an City 710000, China; ^2^Department of Oncology, The First Affiliated Hospital of Xi'an Medical College, Xi'an City 710000, China

## Abstract

**Objective:**

It aimed to explore the diagnostic efficacy of multimodal ultrasound images based on mask region with convolutional neural network (M-RCNN) segmentation algorithm for small liver cancer and analyze the expression of zeste gene enhancer homolog 2 (EZH2) and p57 (P57 Kip2) genes in cancer cells.

**Methods:**

A total of 100 patients suspected of small liver cancer were randomly divided into Doppler group (color Doppler ultrasound examination), contrast group (contrast ultrasound examination), elastic group (ultrasound elastography examination), and multimodal group (combined examination of the three methods), with 25 patients in each group. Images were processed by the M-RCNN segmentation algorithm. The results of the pathological biopsy were used to evaluate the diagnostic efficacy of the four methods. The liver tissues were then extracted and divided into observation group 1 (lesion tissue specimen), observation group 2 (liver tissue around cancer lesion), and control group (normal liver tissue), and the expression activities of EZH2 and p57 genes in the three groups were analyzed.

**Results:**

The accuracy of M-RCNN (97.23%) and average precision (AP) (71.90%) were higher than other methods (*P* < 0.05). Sensitivity (88.87%), specific degree of consistency (90.91%), accuracy (89.47%), and consistence (0.68) of the multimodal group were better than the other three groups (*P* < 0.05). Low and medium differentiated cancer tissues had an irregular shape, unclear boundary, uneven internal echo, unchanged/enhanced posterior echo, blood flow level 1∼2, elastic score 4∼5, and enhancement mode fast in and fast out. The positive expression rate of EZH2 in observation group 1 (75.95%) was higher than that in the other two groups, the positive expression rate of p57 in observation group 1 (80.79%) was lower than that in the other two groups, and the positive expression rate of p57 in the highly differentiated cancer foci (80.79%) was significantly lower than that in the middle and low differentiated cancer foci (*P* < 0.05).

**Conclusions:**

M-RCNN segmentation algorithm had a better segmentation effect. Multimodal ultrasound had a good effect on the benign and malignant diagnosis of small liver cancer and had a high clinical application value. The high expression of EZH2 and the decreased expression of p57 can promote the occurrence of small hepatocellular carcinoma, and the deficiency of the P57 gene was related to the low differentiation of cancer cells.

## 1. Introduction

Liver cancer, one of the most common malignant tumors in clinical practice, has a high incidence and mortality, which poses a great threat to people's life and health [1, 2]. During the occurrence of liver cancer, the expressions of enhancer of zeste homolog 2 (EZH2) [3] and p57 gene [4] of flies would change to some extent. EZH2 is an important member of the poly comb group gene family. Studies have found that EZH2 has high expression activity in a variety of cancer diseases with high incidence, such as breast cancer, stomach cancer, bladder cancer, and prostate cancer [5–8]. The p57 gene, also known as the p57 Kip2 gene, belongs to CDK inhibitors (CKIs), which can reduce the activity of cyclin-dependent kinase (CDK), so as to achieve the purpose of inhibiting the proliferation of cancer cells [9, 10]. In hepatocellular carcinoma, the expression activity of the two genes has a certain influence on the development of cancer foci. This point was analyzed in this study. In liver cancer, small liver cancer is difficult to diagnose because there are no obvious symptoms and signs. However, if timely discovery and effective treatment can be obtained, the prognosis is relatively good, with a high surgical resection rate and a 5-year postoperative survival rate [11, 12]. Therefore, early detection and early treatment of small liver cancer are very necessary to reduce mortality.

Clinically, the diagnostic method for small liver cancer is mainly pathological diagnosis, which belongs to the gold standard for small liver cancer diagnosis [13]. However, the diagnosis method is basically after the patient's surgical treatment, and the diagnosis method used before surgery is imaging technology. Ultrasound examination technology has no radiation, is relatively cheap, safe, noninvasive, high resolution, and can carry out real-time dynamic detection, so it has become the preferred method in clinical practice [14]. In recent years, ultrasound technology has been rapidly developed, a variety of ultrasound technologies endlessly emerge in, such as elastic imaging, contrast ultrasound, and Doppler ultrasound technology. With the rich development of ultrasound technology, the diagnostic capability of ultrasound is further improved. Multimodal ultrasound mode is proposed, that is, the joint application of multiple ultrasound technologies makes a single technology complementary [15]. In an ultrasound examination, the assessment of the scope of the lesion requires the physician's visual observation, but often there is an error. Nowadays, with the extensive application of deep learning algorithms in the field of imaging and the large scale of datasets, experts have proposed the automatic segmentation technology of lesions [16]. However, there are ambiguity and artifacts in ultrasonic images due to low accuracy and instability, which are not conducive to image recognition and segmentation [17]. Therefore, experts proposed to use inception network architecture to accurately extract the noise from high-noise ultrasound images and then used data enhancement and an adaptive median filtering algorithm to enhance the stability of segmentation performance to obtain accurate segmentation images of lesions [18]. After research, the method has achieved good results. The segmentation algorithm is called mask region with convolutional neural network (M-RCNN) segmentation algorithm. However, there are few clinical studies on the application of the above segmentation algorithms in the segmentation of small liver cancer lesions.

In summary, patients suspected to have small liver cancer were taken as the research objects, and multimodal ultrasound images based on the M-RCNN segmentation algorithm were used for examination and diagnosis. The diagnostic efficacy was evaluated based on pathological examination results, and the tissues of patients with small liver cancer and normal patients were examined, to analyze the clinical significance of EZH2 and p57 gene expressions, so as to provide more scientific and effective methods and research basis for the diagnosis and treatment of small liver cancer.

## 2. Methods

### 2.1. Study Object and Grouping

A total of 100 patients with suspected small liver cancer treated in our hospital from April 2019 to April 2021 were randomly selected as the research objects. There were 64 male patients and 36 female patients. The patients' age ranged from 24 to 69 years old, with an average age of (45.24 ± 10.13) years old. There was a single lesion found in 74 cases and multiple lesions in 26 cases. The diameter of the lesions ranged from 0.80 cm to 3.00 cm, with an average diameter of (2.13 ± 0.55) cm. A total of 100 patients were divided into four groups by the random number table method, and they were divided into four groups according to the examination methods: Doppler group, contrast group, elastic group, and multimodal group, with 25 patients in each group. Patients in the Doppler group were mainly diagnosed by combining the results of color Doppler ultrasound. Contrast-enhanced ultrasound (CEUS) was used for diagnosis in the contrast group. The elastic group was examined and diagnosed by ultrasonic elastic imaging. In the multimodal group, three ultrasound methods were combined for diagnosis. The ultrasound images of patients in the four groups were processed by the M-RCNN segmentation algorithm. Then, the results of pathological tissue biopsy were used as the gold standard to evaluate the diagnostic efficacy of the four methods. This study had been approved by the relevant medical ethics committee. All patients voluntarily participated and signed informed consent.

Inclusion criteria were as follows: (i) patients with a history of chronic hepatitis B/C; (ii) all patients were examined for the first time and had not received any other symptomatic treatment before; (iii) all patients were over 18 years old; (iv) ultrasound examination was performed for all patients, and the total diameter of the lesions was no more than 3 cm; and (v) all patients had no family history of cancer.

Exclusion criteria were as follows: (i) patients with intrahepatic and intrahepatic metastasis; (ii) female patients in pregnancy or lactation; (iii) patients with malignant tumors at other sites; and (iv) patients with consciousness disorders.

### 2.2. Tissue Specimens and Grouping

When the patient was biopsied, normal liver tissue around the lesion was extracted. The liver tissue samples of patients diagnosed with small hepatocellular carcinoma were prepared, fixed with 40 g/L formaldehyde, embedded in paraffin, and cut as 4 *μ*m thick × continuous section. Normal liver tissue (noncancerous liver disease surgical specimens or necrotic specimens) was collected from 39 patients as the control group. The lesion tissue samples of patients selected in this study were set as observation group 1, and the liver tissue samples around the tumor were set as observation group 2. Then, the expression activities of EZH2 and p57 genes in liver tissues of the three groups were analyzed.

### 2.3. Ultrasound Examination

#### 2.3.1. Inspection Methods

The instrument was a color ultrasonic examination system (model–HI VSION Preirus, Hitachi). Equipment and parameters were set as follows: probe–convex array, scanning frequency was 3–5 MHz. Probe–high-frequency linear array was used, and the scanning frequency was 5–10 MHz. Scanning methods were that the liver was scanned by conventional two-dimensional ultrasound, and the location, number, size, and boundary of the liver lesions were observed. Later, Doppler ultrasound mode, ultrasound elastography mode, and CEUS were used for specific examinations (Figure 1).

#### 2.3.2. Assessment Methods

Doppler ultrasound mode mainly evaluated the grade of blood flow signal of cancer foci to diagnose benign and malignant lesions. The diagnostic methods were as follows: benign lesion was grade 0∼1 blood flow signal, and grade 2 to 3 indicated malignant lesion. Elastic ultrasound imaging mode was mainly used to evaluate the benign and malignant lesions according to the color display fraction of the image. The diagnostic methods were as follows: lesions with a score of 1–3 suggested benign, while lesions with a score of 4–5 suggested malignant. CEUS was mainly used to judge benign and malignant lesions by the characteristics of different enhancement stages. Arterial phase enhancement features were noncharacteristic enhancement, nonenhancement, and enhancement. Clearance characteristics of delayed period and portal vein stage included noncharacteristic clearance, no clearance, and clearance. The diagnostic method was that the lesions not observed were treated as unenhanced, uncleared, and negative diagnosis, or otherwise, positive diagnosis. The evaluation method of multimodal ultrasound was as follows. If the evaluation results of the above single ultrasound were all malignant, the diagnosis of multimodal ultrasound was also malignant. If one of the results was benign, the diagnosis of multimodal ultrasound was also benign. The above ultrasound images were jointly diagnosed by two ultrasound doctors with ≥5a working experience. If the diagnosis results were different, the diagnosis opinions should be unified through discussion and analysis of the department.

### 2.4. M-RCNN Segmentation Algorithm

For this study, inception network structure [19] was used to extract features of ultrasonic images and ReLU was used as the activation function [20]. The key point of inception block network structure was searching for dense structures in the image and to fit local sparse structure malformations. Therefore, the network removed the whole connection layer and combined the clustering thinking, which not only increased the width of the network but also improved the adaptability of the network to multiple scales. Generally speaking, there are complex noises in original images, so it is difficult to extract and segment the features of images. Thus, before the segmentation of the graph, it is necessary to denoise the graph. An adaptive median filter was used for image denoising.

The effect of the adaptive median filter on superposition and long-tail noise removal is very obvious. Compared with the conventional median filtering algorithm, the algorithm can adjust the size of the window through the initial setting so that the details of the signal can be completely saved. It is supposed that *R*_*xy*_ is a filtered window, *m* × *n* is the size of the window, and *m* and *n* satisfy the following requirements, where *N* is any natural number.

(1) $$\begin{array}{c} m,n\in 2N+1. \end{array}$$

Then, the minimum value in the value of the filtering window is set to *Z*_min_, the maximum value is set to *Z*_max_, the median value is set to *Z*_med_, the arbitrary value is set to *Z*_*xy*_, and the maximum size allowed by the filtering window is set to *S*_max_. Since the structure of the adaptive median filter consists of two parts, namely, the first layer (Level A) and the second layer (Level B), the expression of Level A layer can be obtained as follows:

(2) $$\begin{array}{c} A_{1}=Z_{\text{med}}-Z_{\min},\\ A_{2}=-Z_{\max}-Z_{\text{med}}. \end{array}$$

When both *A*_1_ and *A*_2_ are greater than 0, the calculation of Level B layer shall be carried out. Otherwise, the filtering window shall be enlarged, and the calculation of Level A layer shall be repeated within the maximum size *S*_max_ allowed by the filtering window until *A*_1_ and *A*_2_ are greater than 0. If the target result cannot be achieved within the range of *S*_max_, the output is directly set to any value *Z*_*xy*_.

Level *B* is expressed as follows:

(3) $$\begin{array}{c} B_{1}=Z_{xy}-Z_{\min},\\ B_{2}=-Z_{\min}-Z_{xy}. \end{array}$$

When both *B*_1_ and *B*_2_ are greater than 0, any value *Z*_*xy*_ is directly output. Instead, the median number *Z*_med_ is output.

To effectively reduce the training error and generalization error, the method of data enhancement is used to optimize the target image, and the training loss of the model converges to the best range. Common data enhancement methods include clipping, zooming, rotation, and brightness and contrast adjustment. Through data enhancement, the parameters and quantity of training data can be increased.

Part of ultrasonic images are selected, and the images are labeled (manually segmented) by a number of experienced ultrasound doctors. The group of data with the highest reliability calculated by the coefficient of volumetric overlap error (VOE) [21] is used as the gold standard for the detection of segmentation results.

(4) $$\begin{array}{c} \text{VOE}=1-\frac{V_{\text{Dr}.x}\cap V_{\text{Dr}.y}}{V_{\text{Dr}.x}\cup V_{\text{Dr}.y}}, \end{array}$$

*V*_Dr.*x*_ refers to the segmentation results marked by doctor *x*. *V*_Dr.*y*_ refers to the segmentation result that the doctor *y* noted.

The specific evaluation of segmentation effect combines chaotic matrix [22], a conventional evaluation index, with evaluation indexes such as calculation accuracy, accuracy, and recall rate. After calculation, average precision (AP) [23], area under the precision-recall curve of a certain threshold, and accuracy are used to evaluate the results of this study. The specific calculation method is as follows:

(5) $$\begin{array}{c} \text{Accuracy}=\frac{\text{TP}+\text{TN}}{\text{TP}+\text{FP}+\text{FN}+\text{TN}},\\ \text{Precision}=\frac{\text{TP}}{\text{TP}+\text{FP}},\\ \text{Recall}=\frac{\text{TP}}{\text{TP}+\text{FN}},\\ \text{AP}=\frac{1}{2}\sum_{i=0}^{n-1}\left({\text{Recall}}_{i+1}-{\text{Recall}}_{i}\right)\left({\text{Precision}}_{i+1}+{\text{Precision}}_{i}\right). \end{array}$$

Accuracy refers to the proportion of true-positive (TP) and true-negative (TN) samples in the total sample number. Precision refers to the percentage of TP in a positive sample of predicted results. Recall refers to the proportion of TP in positive samples that have actually been identified. FN refers to the number of negative samples in the negative sample. *TN* refers to the number of negative samples in the positive sample. The higher the AP result is, the better the segmentation effect is. *i* and *n* indicate that the value range of precision, and recall is within the range of [0,1].

### 2.5. Detection of Specimens

Immunohistochemical assay [24] was used to detect the expression activities of EZH2 and p57. The selected materials included EZH2/p57 mouse anti-human monoclonal antibody/biotin detection kit/DAB chromogenic agent (Beijing Zhongshan Jinqiao Biotechnology Co., Ltd.), mouse anti-human PCNA monoclonal Antibody (M12) (Abnova, China), Elivision two-step detection reagent (Fuzhou Maixin Biotechnology Development Co., Ltd.), and cell apoptosis in situ detection kit (Abcam Biotechnology Co., Ltd.). The EZH2 detection procedure referred to dewaxing and hydration of the paraffin section first and then repairing the specimen with high antigen pressure. Subsequently, the tissue samples were treated with 3% H_2_O_2_ to block endogenous peroxidase, and the primary antibody was dropped after 20 min and incubated at 37 °C for 1h. Then, polymer adjuvant was added and incubated for 20 min. Horseradish enzyme-labeled sheep anti-rabbit IgG polymer was added. After incubation for 20 min, DAB was used for chromogenic treatment, hematoxylin was redyed, dehydration was transparent, and tablets were sealed.

The p57 detection steps were as follows: dewaxed and hydrated sections were treated with 3% H_2_O_2_, placed in citric acid buffer with a pH value of 6.0, and underwent high-temperature and high-pressure antigen thermal repair for 5 min. It was taken out and cooled at 37°C, incubated with sheep serum for 30 min, and added with primary antibodies (p57 and PCNA antibodies), which was placed in a wet box and incubated at a constant temperature of 37°C for 2 h. Then, 50 *μ*L of the two reagents A and B each in the two-step detection kit was successively added in two times and incubated at room temperature for 1 h. In the same way, color was developed and redyed. Then, p57 detection required differentiation of hydrochloric acid and alcohol, dehydration and transparency, and neutral gum sealing.

The observation method was double-blind [25], that is, each specimen was randomly observed in five high-power fields (×400, counting 120 tumor cells/each field). The semiquantitative integral method [26] and the percentage score of positive cells were used for evaluation. When the product of the two scores was more than three, the result was positive.

### 2.6. Observed Indexes

Based on pathological diagnosis results, the sensitivity, specificity, and accuracy of the four diagnostic methods were calculated and compared. Edmondson-Steiner method was used to classify small hepatocellular carcinoma into highly differentiated grade I, moderately differentiated grade II, and poorly differentiated grade III and IV. The three grades of differentiation and their corresponding grades were observed to illustrate the ultrasound signs of patients in the multimodal group under different pathological grades.

The positive expressions of EZH2 and p57 in liver tissue samples of the three groups were observed, and the positive expressions of EZH2 and p57 in different pathological differentiation grades were observed.

### 2.7. Statistical Methods

SPSS 25.0 was used for data analysis. The chi-square test or Fisher's exact probability method was used to analyze the difference of multimodal ultrasound features between benign and malignant nodules and small liver cancer with different pathological grades. Measurement data were expressed as *x* ± *s*. Kappa test was used to analyze the consistency of diagnosis results of small liver cancer by Doppler ultrasound, ultrasound elastography, CEUS, and multimodal ultrasound. If 0.70 > Kappa ≥ 0.45, the diagnostic consistency was good. Kappa ≥ 0.7 indicated satisfactory diagnostic consistency. Kappa < 0.45 indicated poor diagnostic consistency, and *P* < 0.05 indicated a statistically significant difference.

## 3. Results

### 3.1. Segmentation Results

The effectiveness of the adopted M-RCNN segmentation algorithm was compared with that of the inception network segmentation algorithm alone (IN), IN optimized only by adaptive median filtering (M-IN), and IN optimized only by data enhancement (S-IN). The results of accuracy and AP are shown in Figure 2. The segmentation accuracies of M-RCNN, IN, M-IN, and S-IN were 97.23%, 87.34%, 90.46%, and 89.67%, respectively. The AP values were 71.90%, 60.88%, 63.78%, and 62.91%, respectively. The accuracies of M-RCNN and AP were significantly higher than the other three segmentation methods (*P* < 0.05).  Figure 3 shows the segmentation effect diagrams of four algorithms for different ultrasonic images, which indicated that M-RCNN segmentation was relatively more detailed.

### 3.2. Comparison of General Clinical Data

The distribution of gender, age, and course of disease were compared among the four groups. In terms of gender and mean age distribution, male patients in the Doppler group, contrast group, elastic group, and multimodal group accounted for 21.88% (14/64), 26.56% (17/64), 25.00% (16/64), and 26.56% (17/64), respectively. Female patients accounted for 27.78% (10/36), 25.00% (9/36), 22.22% (8/36), and 25.00% (9/36), respectively. The mean ages were (44.94 ± 10.44) years, (45.99 ± 11.22) years, (43.24 ± 10.67) years, and (46.14 ± 9.89) years, respectively. After comparison, there was no significant difference in the distribution and average age of male and female patients in the four groups (*P* > 0.05), as presented in Figure 4. In terms of the distribution of the number and mean diameter of lesions, of 74 patients with single lesions, the percentages of Doppler group, contrast group, elastic group, and multimodal group were 25.68% (19/74), 27.03% (20/74), 24.32% (18/74), and 22.97% (17/74), respectively. Of 26 patients with multiple lesions, the proportions of the Doppler group, contrast group, elastic group, and multimodal group were 26.92% (7/26), 23.08% (6/26), 23.08% (6/26), and 26.92% (7/26), respectively. Average diameter was (2.24 + 0.48) cm, (2.01 + 0.59) cm, (2.11–0.57) cm, and (2.14–0.61) cm, respectively. After comparison, there was no significant difference in the number and average diameter distribution of lesions among the four groups (*P* > 0.05, Figure 5).

### 3.3. Diagnosis Effect

A total of 152 foci were found in 100 patients, among which 110 were diagnosed as malignant lesions (79 patients in total). A total of 42 patients were diagnosed as benign, for a total of 21 patients. The results of pathological diagnosis distribution and ultrasonic diagnosis distribution of Doppler group, contrast group, elastic group, and multimodal group are shown in Table 1. The diagnostic sensitivities of the Doppler group, contrast group, elastic group, and multimodal group were 57.69%, 58.06%, 61.54%, and 88.87%, respectively. The specificities were 66.67%, 66.67%, 70.00%, and 90.91%, respectively. The accuracies were 63.16%, 60.00%, 63.89%, and 89.47%, respectively. Kappa values were 0.46, 0.49, 0.48, and 0.68, respectively. Analysis and comparison showed that the multimodal group had better diagnostic sensitivity, specificity, accuracy, and consistency (Kappa) than the other three groups (*P* < 0.05, Figure 6).

### 3.4. Multimodal Ultrasound Features at Different Pathological Grades

According to the statistics, the pathological grading distributions of 110 malignant lesions were 49 (38 cases) with low differentiation, 40 (26 cases) with medium differentiation, and 21 (15 cases) with high differentiation. The signs of multimodal ultrasound images of small liver cancer lesions with different differentiation grades were observed, including shapes, boundaries, internal echoes, posterior echoes, blood flow grading, ultrasonic elastic score, and enhancement mode, as presented in Figure 7. In terms of shape, low and medium differentiation were mainly irregular (79.59%, 70%), and high differentiation was mainly regular (66.67%). In terms of boundary definition, low and middle differentiation were mostly unclear (75.51% and 70.00%), while high differentiation was mostly clear (66.67%). In terms of the uniformity of internal echo, the low and medium differentiation were mainly inhomogeneous (93.88%, 72.5%), and the well-differentiated lesions were mainly homogeneous (66.67%). In terms of whether the posterior echo was enhanced or not, the low and medium differentiation were mostly unchanged/enhanced (89.8% and 72.5%), while the high differentiation lesions had no main features. In terms of blood flow grading, the proportion of low, medium, and high differentiation was higher than that of high differentiation (95.92%, 90.00%, and 66.67%, *P* < 0.05). In terms of ultrasound elastic score, low and medium differentiation were mainly 4–5 points (89.8% and 40%), while high differentiation lesions had no main features. In terms of enhancement mode, the low, medium, and high differentiation were mainly fast in and fast out, but the low and medium differentiation were significantly higher than the high differentiation (83.67%, 80.00% vs. 57.14%) (*P* < 0.05).

### 3.5. Expression of EZH2 Protein and p57 Protein

EZH2 was mainly expressed in the nucleus as brownish yellow granules, while p57 protein was mainly expressed in the cytoplasm or nucleus as brownish or brownish yellow granules, which were distributed in different tissues (Figure 8). The sample numbers of observation group 1 and observation group 2 were the number of small liver cancer patients diagnosed in this study, so the sample numbers were 79. The positive expression rate of EZH2 in observation group 1 (75.95%) was higher than that in observation group 2 and control group (15.19% and 10.26%). The positive expression rate of *p*57 in observation group 1 (40.04%) was higher than that in observation group 2 (79.75%, 94.87%) and control group (*P* < 0.05, Tables 2 and 3).

### 3.6. The Positive Rate of EZH2 and p57 at Different Levels of Pathological Differentiation

There were 38 cases of poorly differentiated foci, 26 cases of moderately differentiated foci, and 15 cases of highly differentiated foci at pathological grade. The expressions of EZH2 and p57 at different differentiation grades were compared. The positive rate of EZH2 expression was 55.26% in poorly differentiated cancer foci, 53.85% in moderately differentiated cancer foci, and 53.33% in highly differentiated cancer foci, with no significant difference (*P* > 0.05). The positive expression rate of p57 was 16.83% in poorly differentiated cancer foci, 20.59% in moderately differentiated cancer foci, and 80.79% in highly differentiated cancer foci. After comparison, it was found that the positive expression rate of p57 in highly differentiated cancer foci was significantly lower than that in medium and low differentiated cancer foci (*P* < 0.05, Figure 9).  Figure 10 shows the expression activity of small liver cancer tissues of different pathological grades. Among them, the expression activity of A2 cancer cells was the highest, and the expression activity of A1 was the lowest.

## 4. Discussion

Abdominal ultrasound has become the preferred method for liver examination because of its high safety and high display of liver structure [27]. However, due to the influence of anatomical sites, operating techniques, experience, and examination instruments and equipment, the accuracy of diagnosis is insufficient [28]. Therefore, multimodal ultrasound emerged, and various single technologies complement each other to improve the diagnostic effect of diseases, especially malignant tumors [29].

Patients suspected of small liver cancer were divided into the Doppler group, control group, elastic group, and multimodal group. The results of pathological diagnosis were used as the gold standard to evaluate the diagnostic effect. The diagnostic sensitivity (88.87% vs. 57.69%, 58.06%, and 61.54%), specificity (90.91% vs. 66.67%, 66.67%, and 70.00%), accuracy (89.47% vs. 63.16%, 60.00%, and 63.89%), and consistency (0.68 vs. 0.46, 0.49, and 0.48) of the multimodal group were better than the other three groups (*P* < 0.05). This is consistent with the results of Hu et al. [30] and Yao et al. [31]. Xiang et al. [32] indicated that multimodal ultrasound has a high effect on benign and malignant diagnosis of breast tumors, which provides support for this study. In addition, multimodal ultrasound showed that the multimodal imaging of poorly differentiated and moderately differentiated cancer tissues mainly showed irregular morphology, unclear boundary, uneven internal echo, unchanged/enhanced posterior echo, blood flow grade 1–2, and ultrasonic elastic score 4–5. Seehawer et al. [33] also proposed that the high aggressiveness of cancer cells would lead to irregular ultrasound images and uneven internal echoes of lesions. In poorly differentiated cancer tissues, the intercellular bridge is not clear, and the nuclear atypia is obvious, while the cell tissue necrosis exists in nuclear division, which leads to the adhesion of surrounding tissues, reducing their activity and tissue elasticity, and increasing their hardness [34]. Deng et al. [35] proposed that vascular density in cancer foci is closely related to the degree of tissue differentiation in cancer foci, and patients with a lower degree of differentiation have higher blood flow grade. It is consistent with the results of this study, which indicates that there are differences in the ultrasound signs of small liver cancer tissues with different pathological grades, and ultrasound examination can be used for the diagnosis of pathological grades.

Expressions of EZH2 and p57 proteins in small liver cancer lesions were studied. The results showed that the positive expression rate of EZH2 in observation group 1 (75.95%) was higher than that in observation group 2 and control group (15.19% and 10.26%), suggesting that abnormal expression of EZH2 was related to the occurrence of small liver cancer. Studies suggested that EZH2 is highly expressed in small liver cancer, which affects the survival rate of patients [36]. Several studies pointed out that EZH2 is significantly (*P* < 0.05) expressed in human hepatocellular carcinoma tissues and cell lines. The positive expression rate of p57 in observation group 1 was lower than that in observation group 2 and control group, suggesting that the insufficient expression of p57 protein was associated with the occurrence of small liver cancer. This was consistent with the research results of Li et al. [37]. Mei et al. [38] also proposed that reduced P57 protein would lead to further development of cancer foci.

To improve the accuracy of this study, the M-RCNN segmentation algorithm was adopted in ultrasonic image processing to improve the display effect of lesions. The results showed that the accuracies of M-RCNN (97.23%) and AP (71.90%) were significantly higher than the other three segmentation methods (*P* < 0.05), indicating that the adopted segmentation algorithm was effective. In addition, it was proposed that the combination of data enhancement and adaptive median filtering has a good optimization effect [39]. The inception network module combining these two methods should be more effective in medical image segmentation processing, which reflects the results of this study, but there are few related studies and further confirmation is needed.

## 5. Conclusion

In this study, multimodal ultrasound images based on the M-RCNN segmentation algorithm were used to examine and diagnose small liver cancer patients, and the diagnostic performance was evaluated. Then, the expressions of EZH2 and p57 genes in cancer cells were studied. The results showed that the M-RCNN segmentation algorithm was more effective in ultrasonic image processing. Multimodal ultrasound had high accuracy in benign and malignant diagnosis of small liver cancer and had high consistency with pathological results, which was of good clinical application value. Both the high expression of EZH2 and the low expression of the p57 gene promoted the occurrence of small hepatocellular carcinoma, and the deficiency of the p57 gene in tumor foci was related to the low differentiation of cancer cells. However, due to the small number of cases in each group, the calculation of the results was not accurate, and the results were not representative enough in this study, which will be corrected in the future study. In conclusion, multimodal ultrasound technology has a good application prospect in the diagnosis of clinical tumor diseases and is worthy of promotion and application.

## Figures and Tables

**Figure 1:** Ultrasonic examination methods.

**Figure 2:** Comparison of accuracy and AP results.

**Figure 3:** Segmentation results.

**Figure 4:** Gender and age distribution.

**Figure 5:** The number and mean diameter distribution of lesions.

**Figure 6:** Comparison of diagnostic effects.

**Figure 7:** Multimodal ultrasound characteristics of different pathological grades. (A-shape, B-boundary, C-internal echo, D-posterior echo, E-blood flow grading, F-ultrasound elastic score, G-enhancement mode, FFFO-fast in and fast out, and FFNO-fast in and no out).

**Figure 8:** Expression of EZH2 and p57 in various liver tissues.

**Figure 9:** Positive rates of EZH2 and p57 at different levels of pathological differentiation.

**Figure 10:** The expression of EZH2 in small liver cancer and adjacent tissues (A1-Adjacent tissue; A2-Highly differentiated; A3-Mediumly differentiated; and A4-Poorly differentiated).

**Table 1:** Statistical diagnosis results of patients in four groups.

Doppler group		Pathological diagnosis (*n* = 38)		Total
		Malignant	Benign	
Doppler ultrasound diagnosis (*n* = 38)	Malignant	16	4	22
	Benign	10	8	18
Total		26	12	38

Contrast group		Pathological diagnosis (*n* = 40)		Total
		Malignant	Benign	
CEUS diagnosis (*n* = 40)	Malignant	18	3	21
	Benign	13	6	19
Total		31	9	40

Elastic group		Pathological diagnosis (*n* = 36)		Total
		Malignant	Benign	
Ultrasound elastography diagnosis (*n* = 36)	Malignant	16	3	19
	Benign	10	7	17
Total		26	10	36

Multimodal group		Pathological diagnosis (*n* = 38)		Total
		Malignant	Benign	
Multimodal ultrasound diagnosis (*n* = 38)	Malignant	24	1	25
	Benign	3	10	13
Total		27	11	38

**Table 2:** Expression of EZH2.

Group		Observation group 1 (*n* = 79)	Observation group 2 (*n* = 79)	Control group (*n* = 79)	*χ* ^2^	*P*

EZH2	Negative	19	67	35	8.23	0.01
	Positive	60	12	4		
*χ* ^2^		8.09			—	
*P*		<0.01				

**Table 3:** Expression of p57.

Group		Observation group 1 (*n* = 79)	Observation group 2 (*n* = 79)	Control group (*n* = 79)	*χ* ^2^	*P*

p57	Negative	49	16	2	8.13	0.01
	Positive	34	63	37		
*χ* ^2^		8.01			—	
*P*		0.01				

## Data Availability

All relevant data are within the manuscript and its Supporting Information files.
